# Optimal Deep-Learning-Enabled Intelligent Decision Support System for SARS-CoV-2 Classification

**DOI:** 10.1155/2022/4130674

**Published:** 2022-01-25

**Authors:** Ashit Kumar Dutta, Nasser Ali Aljarallah, T. Abirami, M. Sundarrajan, Seifedine Kadry, Yunyoung Nam, Chang-Won Jeong

**Affiliations:** ^1^Department of Computer Science and Information Systems, College of Applied Sciences, AlMaarefa University, Ad Diriyah Riyadh 13713, Saudi Arabia; ^2^Department of Business Administration, AlMajmaah University, Saudi Arabia; ^3^AlMaarefa University, Riyadh, Saudi Arabia; ^4^Department of Information Technology, Kongu Engineering College, Erode 638060, India; ^5^Department of Computer Science and Engineering, K. Ramakrishnan College of Engineering, Tiruchirappalli 621112, India; ^6^Department of Applied Data Science, Noroff University College, Kristiansand, Norway; ^7^Department of Computer Science and Engineering, Soonchunhyang University, Asan, Republic of Korea; ^8^Medical Convergence Research Center, Wonkwang University, Iksan, Republic of Korea

## Abstract

Intelligent decision support systems (IDSS) for complex healthcare applications aim to examine a large quantity of complex healthcare data to assist doctors, researchers, pathologists, and other healthcare professionals. A decision support system (DSS) is an intelligent system that provides improved assistance in various stages of health-related disease diagnosis. At the same time, the SARS-CoV-2 infection that causes COVID-19 disease has spread globally from the beginning of 2020. Several research works reported that the imaging pattern based on computed tomography (CT) can be utilized to detect SARS-CoV-2. Earlier identification and detection of the diseases is essential to offer adequate treatment and avoid the severity of the disease. With this motivation, this study develops an efficient deep-learning-based fusion model with swarm intelligence (EDLFM-SI) for SARS-CoV-2 identification. The proposed EDLFM-SI technique aims to detect and classify the SARS-CoV-2 infection or not. Also, the EDLFM-SI technique comprises various processes, namely, data augmentation, preprocessing, feature extraction, and classification. Moreover, a fusion of capsule network (CapsNet) and MobileNet based feature extractors are employed. Besides, a water strider algorithm (WSA) is applied to fine-tune the hyperparameters involved in the DL models. Finally, a cascaded neural network (CNN) classifier is applied for detecting the existence of SARS-CoV-2. In order to showcase the improved performance of the EDLFM-SI technique, a wide range of simulations take place on the COVID-19 CT data set and the SARS-CoV-2 CT scan data set. The simulation outcomes highlighted the supremacy of the EDLFM-SI technique over the recent approaches.

## 1. Introduction

Intelligent decision support systems (IDSS) has become widely used in several applications of healthcare. Internet of things (IoT), wearables, manual data entry, and online sources are some of the instances of complex data sources for IDSS. The data sustained by IDSS significantly helps in the earlier identification of diseases and equivalent treatments. The coronavirus disease 2019 (COVID-19) epidemic, caused by severe acute respiratory syndrome coronavirus 2 (SARS-CoV-2), began in Wuhan city, Hubei province, in December, 2019, and has spread throughout China. COVID-19 is an infectious disease caused by the novel coronavirus named SARS-CoV-2. The virus is extremely infectious, and can be transmitted by indirect or direct contact with diseased persons with respiratory droplets while they cough, sneeze, or even talk [1]. Now, the real-time polymerase chain reaction (RT-PCR) test is the common method used to confirm COVID-19 infection, and with the rapid rise in the number of diseased persons, almost all countries are confronting a shortage of testing kit. Furthermore, RT-PCR testing can have a higher false-negative rate and turnaround times [2]. Therefore, it is appropriate for considering other testing tools for detecting COVID-19 infected people to isolate them and alleviate the pandemic impact on the lives of several people. The chest computed tomography (CT) is an appropriate supplement to RT-PCR testing and plays a role in diagnosing and screening COVID-19 infection. In current works [3], the researchers manually investigated chest CT scans of over thousands of patients and confirmed the helpfulness of chest CT scan in COVID-19 detection with a higher sensitivity rates.

In certain cases, the patient had a negative PCR test at first, but confirmation was depending on their CT results. Additionally, chest CT screening was suggested, while the patient shows compatible symptoms with COVID-19; however, the outcome of its PCR tests is negative [4]. Hence, it is necessary for an automatic detection tool that exploits the current developments in deep learning (DL) and artificial intelligence (AI), as well as the accessibility of CT images to construct AI-based tools to prevent further spreading and expedite the diagnoses method [5]. In order to mitigate the shortage and inefficiency of current tests for COVID-19 infection, various attempts have been dedicated to seeking alternate testing tools [6]. Various researches have exposed that CT scans manifest strong radiological results of COVID-19 and are promising in serving as an accessible and more efficient testing tool because of the wider accessibility of CT devices, which could achieve results at the highest rate. Furthermore, to mitigate the burden of medical specialists from reading CT scans, numerous studies have designed DL algorithms that could automatically interpret CT images and forecast whether the CT is positive for COVID-19 infection. When this work has demonstrated effective outcomes, they have two limitations [7]. Initially, the CT scans data set utilized in this study are not accessible to the public because of security concerns.

Accordingly, their results could not be reproduced, and the trained methods could not be utilized in other hospitals. In addition, the lack of open-sourced annotated COVID-19 CT data sets seriously hinders the development and research of innovative AI tools for precise CT-based testing of COVID-19 infection [8]. Next, this study requires a wide range of CTs at the time of model training to accomplish performances that meet the medical standards. These requirements are practically stringent, and it could not met by several hospitals, particularly under the circumstance that medical experts are very occupied in handing COVID-19 infected patients and do not have time to annotate and collect a huge amount of COVID-19 CT scans.

This study develops an efficient deep-learning-based fusion model with swarm intelligence (EDLFM-SI) for SARS-CoV-2 identification for complex healthcare applications. Moreover, the EDLFM-SI technique comprises a fusion of capsule network (CapsNet) and MobileNet based feature extractors are employed. Furthermore, a water strider algorithm (WSA) is applied to fine-tune the hyperparameters involved in the DL models. Lastly, a cascaded neural network (CNN) classifier is applied to detect the existence of SARS-CoV-2. For examining the enhanced outcomes of the EDLFM-SI technique, a comprehensive experimental analysis is carried out on the COVID-19 CT data set and the SARS-CoV-2 CT scan data set.

The rest of the paper is organized as follows.  Section 2 offers the related works; Section 3 elaborates the proposed model; Section 4 provides the result analysis; and Section 5 draws the conclusions.

## 2. Related Works

This section provides a comprehensive review of existing COVID-19 detection models. Biswas et al. [9] aimed to determine a strong COVID-19 predictive method via chest CT images through effective TL methods. At first, they utilized three typical DL algorithms, such as Xception, VGG-16, and ResNet50, for COVID-19 prediction. Next, they presented a method to integrate the abovementioned pretrained method for the general enhancement of the predictive capacity of the model. Ibrahim et al. [10] proposed a new computer-aided framework (COV-CAF) to categorize the severity level of the disease from three-dimensional CT Volumes. COV-CAF integrates conventional and DL methods. The presented COV-CAF method contains two stages: the preparatory stage and the feature analysis and classification stage. The feature analysis and classification stage integrates fuzzy clustering for feature fusion and automated RoI segmentation.

In Dansana et al. [11], the CNN approach is utilized to binary classification pneumonia-based transformation of Inception_V2, DT, and VGG-19 methods on CT scan and X-ray image data sets that have 360 images. It could gather that fine-tuned VGG-19, Inception_V2, and DT methods show outstanding performances with an increased rate of validation and training accuracy. Wang et al. [12] hypothesized that AI method that could extract certain graphical features of COVID-19 and offer medical diagnoses in advance of the pathogenic test, therefore saving critical time for controlling the disease. They gathered 1,065 CT images of pathogen-confirmed COVID-19 cases and persons who were diagnosed previously with standard COVID-19. They adapted the inception TL method for establishing the model, followed by external and internal validations.

Mei et al. [13] employed AI methods for integrating chest CT results with laboratory testing, medical symptoms, and exposure history to quickly analyze persons with positive for COVID-19. Goel et al. [14] presented a novel architecture for exploiting effective features extracted from the AE and GLCM, integrated with the RF model for the effective and faster diagnosis of COVID-19 with CT images. Mohammed et al. [15] presented an automatic CAD system for COVID-19-based chest X-ray image analyses. It is developed for COVID-19 diagnosis from another ARDS, MERS, and SARS infection. The optimum threshold values for chest images segmentation are deduced by using Li's model and PSI method. Then, Laws' mask is employed in the chest image segmentation for highlighting secondary characteristics. Next, nine distinct vectors of features are extracted from the GLCM of every Laws' mask finding. The ensemble SVM methods are constructed according to the extracted feature vector. Munir et al. [16] presented a DNN method that is trained on the X-ray image of the COVID-19 and standard X-ray images to the COVID-19 diagnosis. Alquzi et al. [17] developed a result to detect persons with COVID-19 from CT images and ML models. This method is depending on a CNN model named EfficientNet.

## 3. The Proposed EDLFM-SI Technique

In this study, an effective EDLFM-SI technique is designed to detect and classify the SARS-CoV-2 infection or not. Also, the EDLFM-SI technique comprises various processes namely data augmentation, preprocessing, fusion-based feature extraction, WSA-based hyperparameter optimization, and CNN-based classification. At the same time, a fusion of CapsNet and MobileNet based feature extractors are employed.  Figure 1 illustrates the overall process of the EDLFM-SI model. The working principle of every process is elaborated in the succeeding sections.

### 3.1. Preprocessing and Data Augmentation

Primarily, median filtering is applied for removing the noise present in the test CT images. Next, data augmentation comprises raising the number of training instances by the transformation of the images with no loss of semantic details. In this study, data augmentation takes place in three ways such as rotation, horizontal flip, and scaling.

### 3.2. Fusion-Based Feature Extraction

At this stage, the fusion-based feature extraction process is employed in which the fusion of MobileNet and CapsNet features is extracted.

#### 3.2.1. MobileNet Model

The MobileNet V2 enhances efficiency of mobile techniques on several tasks and benchmarks and through the spectrum of various technique sizes. The basic principle behind MobileNet technique is the replacement of convolutional layers with depthwise separable convolution blocks where the depthwise convolution layer is trailed by the pointwise convolution layer to create effective feature vectors. It can be much greater than the regular convolutional with around similar outcomes. In MobileNet V2, all the blocks include 1 × 1 development layer from more depthwise and pointwise convolution layers. Different Vl, the pointwise convolution layer of *V*2 recognized as the prediction layer projects information with the maximum amount of channels as to tensor with a considerably minimum amount of channels. MobileNetv2 is based on an inverted residual structure where the residual connections exist among the bottleneck layers. A 1 × 1 expansion convolution layer has increased the amount of channels dependent upon expansion issue from the data previously as it goes to depthwise convolutions. The second novel thing from MobileNet V2's structure block has remaining linking [18]. The remaining linking uses the flow of gradient with networks.

Computation cost is considerably lower than the typical convolution with a compromise in slightly reduced accuracy.

#### 3.2.2. CapsNet Model

For overcoming the limitations of CNN and generating it nearby the cerebral cortex activity framework, Hinton [19] presented a maximum dimension vector named as “capsule” for representing an entity (an object or part of object) with a set of neurons before a single neuron. All the capsules learn an implicit explanation of visual entity that output the probabilities of the entity and the group of “instantiated parameter containing the precise pose (place, size, and orientation), deforming, velocity, albedo, hue, texture, and so on.

The structure of CapsNet has been distinct in other DL techniques. The outcomes of input and output of CapsNets have been vectors whose norm and way demonstrate the existence probabilities and several attributes of entity correspondingly. If the several forecasts have been consistent, the higher level of one capsule is developed actively.  Figure 2 depicts the framework of the CapsNet model. The structure has been shallow with only two convolution layers (Convl, and PrimaryCaps) and one fully connected (FC) layer (EntityCaps). In detail, Convl has the typical convolution layer that alters images to initial features and outcomes to PrimaryCaps with a convolutional filter with a size of 13 × 13 × 256. During the case where the original image is not appropriate to the input of the primary layer of the CapsNet, the rule feature then convolution was implemented.

The second convolution layer generates the equivalent vector framework as input of the capsule layer [20]. The typical convolutional of all output is scalars; however, the convolutional of PrimaryCaps has distinct from the classical one. It is considered 2‐D convolutional of eight distinct weights to the input of 15 × 15 × 256. The third layer (EntityCaps) has been the resultant layer that has nine typical capsules equivalent to nine distinct classes.

A layer of CapsNet has been separated into several computational units called capsules. Consider a capsule *i* with activity neuron *i*, it can be given as capsule *j* for generating activity level *v*_*j*_ of EntityCaps. The propagating and upgrading have been conducted utilizing vectors among PrimaryCaps and EntityCaps. The matrix model was employed to scalar input from all the layers of typical NN that is basically a linear combination of outcomes. The capsule modeling input has been separated into two phases: linear combination as well as routing. The linear combination represents an idea of modeling scalar input with NN that implies processing the connection among two objects from the scene with a visual alteration matrix but maintaining its relative relation. In detail, the linear combination was expressed as follows:

(1) $$\begin{array}{c} {\hat{u}}_{j|i}=u_{i}W_{ij}, \end{array}$$

where $\hat{u}$ refers to the forecast vector created by changing the outcome *u*_*i*_ of the capsule from the layer under by weight *W*_*ij*_. Afterward, during the routing phase, the input vector *s*_*j*_ of the capsule, *j* is determined as follows:

(2) $$\begin{array}{c} s_{j}=\sum_{i}c_{ij}{\hat{u}}_{j|i}, \end{array}$$

where *c*_*ij*_ implies the coupling coefficient defined as the iterative dynamic routing procedure. The routing part comprises a weighted sum of $\hat{u}$ coupling coefficients. The vector output of capsule *j* has computed by implementing a non-linear squashing function produces

(3) $$\begin{array}{c} v_{j}=\frac{{\left\|s_{j}\right\|}^{2}}{1+|{\left\|s_{j}\right\|}^{2}}\frac{s_{j}}{\left\|s_{j}\right\|}.\; \end{array}$$

Noticeably, the capsule activation function essentially suppresses as well as redistributes vector length. Its output has been utilized as probabilities of entity signified as the capsule from the present type. The entire loss function of novel CapsNet has a weighted summation of marginal loss and reconstructing loss. The MSE has utilized from the novel reconstructing loss function that degrades this technique considerably if modeling noisy data.

#### 3.2.3. Fusion Process

Data fusion is employed in many applications of ML and CV methods. Feature fusion is an important task that integrates one or more feature vectors. The proposed method is dependent on feature fusion through entropy. The two vectors are described as follows:

(4) $$\begin{array}{c} {\text{f}}_{\text{CapsNet}1\times n}=\left\{{\text{CapsNet}}_{1\times 1},{\text{CapsNet}}_{1\times 2},{\text{CapsNet}}_{1\times 3},\ldots ,{\text{CapsNet}}_{1\times n}\right\},\\ {\text{f}}_{\text{EfficientNet}191\times m}=\left\{{\text{MobileNet}}_{1\times 1},{\text{MobileNet}}_{1\times 2},{\text{MobileNet}}_{1\times 3},\ldots ,{\text{MobileNet}}_{1\times m}\right\}. \end{array}$$

Besides, the extracted features are integrated into a single vector using the following equation:

(5) $$\begin{array}{c} \text{Fused}{\left(\text{features vector}\right)}_{1\times \text{q}}=\sum_{i=1}^{2}{\text{fCapsNet}}_{1\times \text{n}},{\text{fMobileNet}}_{1\times \text{m}}, \end{array}$$

where *f* represents fused vectors (1 × 1186). The entropy is utilized on features vectors for the selection of optimum features according to the score.

### 3.3. Hyperparameter Optimization

In order to optimally adjust the hyperparameters involved in the fusion model, the WSA is applied to it. The WSA is a population-based method that stimulates succession of water strider bugs, territorial behavior, feeding mechanism, mating style, and intelligent ripple communication. This method is described briefly in the following steps.

#### 3.3.1. Initial Birth

The candidate solution/water strider (WS) is arbitrarily caused in the searching space as follows:

(6) $$\begin{array}{c} WS_{i}^{0}=Lb+\text{rand,}\\ \left(Ub-Lb\right);\;i=1,2,\ldots ,\text{nws}, \end{array}$$

where WS_*i*_^0^ represents the first position of *i*-th WS in the lake (search space). *Lb* and *Ub* represent lower and upper bounds, respectively. rand denotes an arbitrary value in the range of zero and one, and nws indicates the amount of WS_*s*_ (population size). The first position of WS_*s*_ is estimated by an objective function to evaluate the fitness.

#### 3.3.2. Territory Establishment

To determine nt amount of territories, WS_*s*_ is arranged based on their fitness, and nws/nt amount of groups are generated orderly. The *j*-th member of all the groups is allocated to the *j*-th territory, where *j*=1,2,…, nt. Thus, the amount of WS_*s*_ lives in all the territories are equivalent to nws/nt. The position in all the territories with the best and worst fatness is considered female and male (keystone), respectively.

#### 3.3.3. Mating

The male WS transmits ripple to female WS for mating. As the response of females is unknown, a probability *p* is determined for attraction or else repulsion [21]. The *p* is fixed to 0.5. The location of the male WS is upgraded as follows:

(7) $$\begin{array}{c} \left\{\begin{array}{c} {\text{WS}}_{i}^{t+1}={\text{WS}}_{i}^{t}+R.\text{rand;if mating happens }\left(\text{with probability of p}\right),\\ {\text{WS}}_{i}^{t+1}={\text{WS}}_{i}^{t}+R.\left(1+\text{rand}\right);\text{ otherwise.} \end{array}\right. \end{array}$$

The length of *R* is estimated as follows:

(8) $$\begin{array}{c} R={\text{WS}}_{F}^{t-1}-{\text{WS}}_{i}^{t-1}, \end{array}$$

where WS_*i*_^*t*−1^ and WS_*F*_^*t*−1^ denotes the male and female WS in the (*t* − 1)^*th*^ cycle, respectively.

#### 3.3.4. Feeding

Mating expends numerous energies for water strider, and the male WS forages to food afterward mating. During the latter scenario, the male WS move towards the optimal WS of lake (WS) for finding foods based on the following equation:

(9) $$\begin{array}{c} {\text{WS}}_{i}^{t+1}={\text{WS}}_{i}^{t}+2{\text{rand}}^{*}\left({\text{WS}}_{BL}^{t}-{\text{WS}}_{i}^{t}\right). \end{array}$$

#### 3.3.5. Death and Succession

In the novel location, the male *WS* could not find food; it would pass away; and a novel *WS* would replace it as follows:

(10) $$\begin{array}{c} {\text{WS}}_{i}^{t+1}={\text{Lb}}_{j}^{t}+{\text{rand}}^{*}\left({\text{Ub}}_{j}^{t}-{\text{Lb}}_{j}^{t}\right), \end{array}$$

where Ub_*j*_^*t*^ and Lb_*j*_ are the maximal and minimal values of WS^†^*s* located inside the *j*-th territory.

#### 3.3.6. WSA Termination

When the end criteria are met, the process would return to the mating step for a novel loop. Now, the maximum amount of function evaluation (MaxNFEs) is considered an end criterion.

### 3.4. CNN-Based Classification

Finally, the features are fed into the CNN model to allot the classes that exist in it. The perceptron linking that has been designed among the input and output has a procedure of direct relation, but FFNN linked generated among input and output was an indirect connection. The link was non-linear from shape with activation function from the hidden layer. When the link generated on perceptron and multilayer network has been joined, afterward, the network with direct link among the input and output layers is created. The network generated in this linking design was named CNN. The formulas are created in the CNN technique that is expressed as follows:

(11) $$\begin{array}{c} y=\sum_{i=1}^{n}f^{i}\omega_{i}^{i}x_{i}+f^{o}\left(\sum_{j=1}^{k}\omega_{j}^{o}f_{j}^{h}\left(\sum_{i=1}^{n}\omega_{ji}^{h}x_{i}\right)\right)\;, \end{array}$$

where *f* refers to the activation function in the input-output layers and *ω*_*i*_^*i*^ implies the weight in the input-output layers [22]. When the bias has more than the input layers and activation function of all the neurons from the hidden layer is *f*^*h*^, then

(12) $$\begin{array}{c} y=\sum_{i=1}^{n}f^{i}\omega_{i}^{i}x_{i}f^{o}\left(\omega^{b}+\sum_{j=1}^{k}\omega_{j}^{o}f\left(\omega_{j}^{b}+\sum_{j=1}^{k}\omega_{j}^{o}f_{j}^{h}\right)\right)\;. \end{array}$$

During this case, the CFNN technique was executed from the time sequences data. So the neurons from the input layer are the delays of time sequences data *X*_*t*−1_, *X*_*t*−2_,…, *X*_*t*−*p*_, but the output has the present data *X*_*t*_.

## 4. Performance Validation

### 4.1. Implementation Data

The experimental validation of the EDLFM-SI technique takes place using two benchmark data set, namely, SARS-CoV-2 CT scan [23] and COVID-19 CT [24, 25] data sets. The former contains a set of 2,482 CT scans with 1,252 scans under SARS-CoV-2 and 1,230 scans under other lung diseases. The next data set includes 746 CT images, with 349 CT images under COVID-19 and 397 CT images under non-COVID-19. Few sample images are demonstrated in Figure 3.

### 4.2. Result Analysis on SARS-CoV-2 CT Scan Data Set

Figure 4 demonstrates the confusion matrices produced by the EDLFM-SI technique on test data set-1. The results exhibited that the EDLFM-SI technique has identified the COVID-19 and non-COVID-19 images correctly under all runs. For instance, with run-1, the EDLFM-SI technique has classified 1,234 images into COIVD-19 and 1,214 images into non-COVID-19. At the same time, with run-4, the EDLFM-SI approach has classified 1,241 images into COIVD-19 and 1,214 images into non-COVID-19. Followed by, with run-6, the EDLFM-SI method has classified 1,237 images into COIVD-19 and 1,216 images into non-COVID-19. Moreover, with run-8, the EDLFM-SI system has classified 1,236 images into COIVD-19 and 1,215 images into non-COVID-19. Furthermore, with run-10, the EDLFM-SI methodology has classified 1,238 images into COIVD-19 and 1,218 images into non-COVID-19.

Table 1 and Figure 5 provide the overall COVID-19 classification outcomes analysis of the EDLFM-SI technique on data set-1. The table depicted that the EDLFM-SI technique has the ability to classify images under all runs. For instance, with run-1, the EDLFM-SI technique has gained increased pre_*n*_, sen_*y*_, spe_*y*_, acc_*y*_, and *F*_score_ of 0.9872, 0.9856, 0.9870, 0.9863, and 0.9864, respectively. Along with that, with run-2, the EDLFM-SI system has reached enhanced pre_*n*_, sen_*y*_, spe_*y*_, acc_*y*_, and *F*_score_ of 0.9888, 0.9904, 0.9886, 0.9895, and 0.9896, respectively. In line with that, with run-6, the EDLFM-SI methodology has attained improved pre_*n*_, sen_*y*_, spe_*y*_, acc_*y*_, and *F*_score_ of 0.9888, 0.9880, 0.9886, 0.9883, and 0.9884, respectively. Followed by that, with run-8, the EDLFM-SI technique has gained increased pre_*n*_, sen_*y*_, spe_*y*_, acc_*y*_, and *F*_score_ of 0.9880, 0.9872, 0.9878, 0.9875, and 0.9876, respectively. Lastly, with run-10, the EDLFM-SI approach has achieved higher pre_*n*_, sen_*y*_, spe_*y*_, acc_*y*_, and *F*_score_ of 0.9904, 0.9888, 0.9902, 0.9895, and 0.9896, respectively.

Figure 6 showcases the accuracy graph analysis of the EDLFM-SI technique on the test data set 1. The figure revealed that the EDLFM-SI technique has resulted in maximum training and validation accuracies. It is observed that the EDLFM-SI technique has accomplished increased validation accuracy compared to training accuracy.

Next, the loss graph analysis of the EDLFM-SI technique under data set-1 takes place in Figure 7. The figure reported that the EDLFM-SI technique has attained minimal training and validation losses. It is also noticeable that the EDLFM-SI technique has resulted in reduced validation loss over the training loss.

A detailed comparative results analysis of the EDLFM-SI technique with recent techniques takes place on data set-1 in Table 2 and Figure 8. The figure shows that the DT model has gained poor outcomes with the lower classification. At the same time, the GN, VGG-16, RN, and AN models have reached moderately closer classification performance. Along with that, the xDNN model has accomplished reasonable classification performance over the other techniques. At last, the proposed EDLFM-SI technique has outperformed the other methods with the maximum pre_*n*_, sen_*y*_, acc_*y*_, and *F*_score_ of 0.9904, 0.9920, 0.9899, and 0.9900, respectively.

### 4.3. Results Analysis on COVID-19 CT Data Set

Figure 9 exhibits the confusion matrices formed by the EDLFM-SI system on the test data set-2. The outcomes showcased that the EDLFM-SI manner has identified the COVID-19 and non-COVID-19 images correctly under all runs.

For sample, with run-1, the EDLFM-SI scheme has classified 331 images into COIVD-19 and 381 images into non-COVID-19. Likewise, with run-4, the EDLFM-SI algorithm has classified 335 images into COIVD-19 and 382 images into non-COVID-19. Similarly, with run-6, the EDLFM-SI technique has classified 333 images into COIVD-19 and 378 images into non-COVID-19. In addition, with run-8, the EDLFM-SI method has classified 332 images into COIVD-19 and 377 images into non-COVID-19. At last, with run-10, the EDLFM-SI approach has classified 331 images into COIVD-19 and 383 images into non-COVID-19.

Table 3 and Figure 10 offer the overall COVID-19 classification outcomes analysis of the EDLFM-SI approach on data set-2. The table outperformed that the EDLFM-SI system has the ability to classify images in all runs. For instance, with run-1, the EDLFM-SI approach has attained maximal pre_*n*_, sen_*y*_, spe_*y*_, acc_*y*_, and *F*_score_ of 0.9539, 0.9484, 0.9597, 0.9544, and 0.9511, respectively. At the same time, with run-4, the EDLFM-SI methodology has attained superior pre_*n*_, sen_*y*_, spe_*y*_, acc_*y*_, and *F*_score_ of 0.9571, 0.9599, 0.9622, 0.9611, and 0.9585, respectively. Besides, with run-6, the EDLFM-SI system has gained maximum pre_*n*_, sen_*y*_, spe_*y*_, acc_*y*_, and *F*_score_ of 0.9460, 0.9542, 0.9521, 0.9531, and 0.9501, respectively. Moreover, with run-8, the EDLFM-SI technique has gained higher pre_*n*_, sen_*y*_, spe_*y*_, acc_*y*_, and *F*_score_ of 0.9432, 0.9513, 0.9496, 0.9517, and 0.9487, respectively. Eventually, with run-10, the EDLFM-SI methodology has gained improved pre_*n*_, sen_*y*_, spe_*y*_, acc_*y*_, and *F*_score_ of 0.9594, 0.9484, 0.9647, 0.9571, and 0.9539, respectively.

Figure 11 illustrates the accuracy graph analysis of the EDLFM-SI approach on the test data set 2. From the figure, it is obvious that the EDLFM-SI technique has resulted in maximal training and validation accuracies. It can be clear that the EDLFM-SI technique has accomplished increased validation accuracy related to training accuracy.

Then, the loss graph analysis of the EDLFM-SI approach on the test data set-2 takes place in Figure 12. The figure stated that the EDLFM-SI system has reached lesser training and validation losses. It can be also obvious that the EDLFM-SI methodology has resulted in decreased validation loss over the training loss.

A brief comparative outcomes analysis of the EDLFM-SI approach with recent systems takes place on data set-2 in Table 4 and Figure 13. The figure demonstrated that the Xception manner has attained worse results with minimum classification. Simultaneously, the DN-121, InceptionV3, RN-101, and DN-169 methods have obtained moderately closer classification performance. Also, the DN-201 model has accomplished reasonable classification performance over the other techniques. At last, the presented EDLFM-SI algorithm has outperformed the other methodologies with the maximal pre_*n*_, sen_*y*_, acc_*y*_, and *F*_score_ of 0.9599, 0.9599, 0.9625, and 0.9060, respectively.

By looking into the detailed tables and figures, it is obvious that the EDLFM-SI technique has resulted in improved COVID-19 detection and classification performance over the recent methods.

## 5. Conclusion

In this study, an effective EDLFM-SI technique is designed to detect and classify the SARS-CoV-2 infection for complex healthcare applications. Also, the EDLFM-SI technique comprises various processes, namely, data augmentation, preprocessing, fusion-based feature extraction, WSA-based hyperparameter optimization, and CNN-based classification. The fusion-based feature extraction process is employed in which the fusion of MobileNet and CapsNet features is extracted. To optimally adjust the hyperparameters involved in the fusion model, the WSA was executed to it. Finally, the features are fed into the CNN model to allot the classes that exist in it. For examining the enhanced outcomes of the EDLFM-SI technique, a comprehensive experimental analysis is carried out on the COVID-19 CT data set and the SARS-CoV-2 CT scan data set. The simulation outcomes highlighted the supremacy of the EDLFM-SI technique over the recent approaches. As a part of the future scope, the classification performance of the proposed EDLFM-SI technique can be employed for SARS-CoV-2 detection by the use of hybrid metaheuristic-based optimization algorithms.

## Figures and Tables

**Figure 1:** Overall block diagram of EDLFM-SI model.

**Figure 2:** Structure of the CapsNet model.

**Figure 3:** Sample images.

**Figure 4:** Confusion matrix of EDLFM-SI model under data set-1: (a) run-1, (b) run-2, (c) run-3, (d) run-4, (e) run-5, (f) run-6, (g) run-7, (h) run-8, (i) run-9, and (j) run-10.

**Figure 5:** Result analysis of EDLFM-SI model under data set-1.

**Figure 6:** Accuracy analysis of EDLFM-SI model under data set-1.

**Figure 7:** Loss analysis of EDLFM-SI model under data set-1.

**Figure 8:** Comparative analysis of EDLFM-SI model under data set-1.

**Figure 9:** Confusion matrix analysis of EDLFM-SI model under data set-2: (a) run-1, (b) run-2, (c) run-3, (d) run-4, (e) run-5, (f) run-6, (g) run-7, (h) run-8, (i) run-9, and (j) run-10.

**Figure 10:** Result analysis of EDLFM-SI model under data set-2.

**Figure 11:** Accuracy analysis of EDLFM-SI model under data set-2.

**Figure 12:** Loss analysis of EDLFM-SI model under data set-2.

**Figure 13:** Comparative analysis of EDLFM-SI model under data set-2.

**Table 1:** Result analysis of EDLFM-SI model with distinct measures under data set-1.

No. of runs	Precision	Sensitivity	Specificity	Accuracy	F-score
Run-1	0.9872	0.9856	0.9870	0.9863	0.9864
Run-2	0.9888	0.9904	0.9886	0.9895	0.9896
Run-3	0.9880	0.9880	0.9878	0.9879	0.9880
Run-4	0.9873	0.9912	0.9870	0.9891	0.9892
Run-5	0.9881	0.9920	0.9878	0.9899	0.9900
Run-6	0.9888	0.9880	0.9886	0.9883	0.9884
Run-7	0.9864	0.9864	0.9862	0.9863	0.9864
Run-8	0.9880	0.9872	0.9878	0.9875	0.9876
Run-9	0.9904	0.9872	0.9902	0.9887	0.9888
Run-10	0.9904	0.9888	0.9902	0.9895	0.9896
Average	0.9883	0.9885	0.9881	0.9883	0.9884

**Table 2:** Comparative analysis of EDLFM-SI model with existing approaches under data set-1.

Methods	Precision	Sensitivity	Accuracy	*F*-score
EDLFM-SI	0.9904	0.9920	0.9899	0.9900
xDNN model	0.0916	0.9553	0.9738	0.9731
RN model	0.9300	0.9715	0.9496	0.9503
GN model	0.9020	0.9350	0.9173	0.9182
VGG-16	0.9402	0.9543	0.9496	0.9497
AN model	0.9498	0.9228	0.9375	0.9361
DT model	0.7681	0.8313	0.7944	0.7984

**Table 3:** Result analysis of EDLFM-SI model under data set-2.

No. of runs	Precision	Sensitivity	Specificity	Accuracy	*F*-score
Run-1	0.9539	0.9484	0.9597	0.9544	0.9511
Run-2	0.9598	0.9570	0.9647	0.9611	0.9584
Run-3	0.9536	0.9427	0.9597	0.9517	0.9481
Run-4	0.9571	0.9599	0.9622	0.9611	0.9585
Run-5	0.9599	0.9599	0.9647	0.9625	0.9599
Run-6	0.9460	0.9542	0.9521	0.9531	0.9501
Run-7	0.9433	0.9542	0.9496	0.9517	0.9487
Run-8	0.9432	0.9513	0.9496	0.9504	0.9472
Run-9	0.9594	0.9484	0.9647	0.9571	0.9539
Run-10	0.9594	0.9484	0.9647	0.9571	0.9539
Average	0.9536	0.9524	0.9592	0.9560	0.9530

**Table 4:** Comparative analysis of EDLFM-SI model with existing approaches under data set-2.

Methods	Precision	Sensitivity	Accuracy	*F*-score
EDLFM-SI	0.9599	0.9599	0.9625	0.9599
RN-101 model	0.8810	0.9310	0.9090	0.9060
InceptionV3	0.8770	0.9000	0.8940	0.8880
Xception	0.8730	0.8830	0.8850	0.8770
DN-121 model	0.8760	0.8880	0.8890	0.8820
DN-169 model	0.8810	0.9370	0.9120	0.9080
DN-201 model	0.9130	0.9370	0.9290	0.9250

## Data Availability

The data set used in this paper is publicly available at the following link: https://www.kaggle.com/plameneduardo/sarscov2-ctscan-dataset and https://github.com/UCSD-AI4H/COVID-CT.
